The article "FOXM1 Promotes Drug Resistance in Cervical Cancer Cells by Regulating ABCC5 Gene Transcription" was published in 2022. Journal: Biomed Res Int.

# FOXM1 Promotes Drug Resistance in Cervical Cancer Cells by Regulating ABCC5 Gene Transcription

**DOI:** 10.1155/2022/3032590

**Published:** 2022-01-31

**Authors:** Youxiang Hou, Zhanfei Dong, Wei Zhong, Linglong Yin, Xiong Li, Gulina Kuerban, He Huang

**Affiliations:** ^1^Department of Radiation Oncology, The Affiliated Cancer Hospital of Xinjiang Medical University, 789 Suzhou Dong Jie, Xinshi District, Urumqi, Xinjiang 86830000, China; ^2^Department of Nuclear Medicine, The Affiliated Cancer Hospital of Xinjiang Medical University, 789 Suzhou Dong Jie, Xinshi District, Urumqi, Xinjiang 86830000, China; ^3^School of Integrative Pharmacy, Institute of Integrative Pharmaceutical Research, Guangdong Pharmaceutical University, 280 Waihuandong Rd, Panyu District, Guangzhou, Guangdong 86510000, China; ^4^Department of Histology and Embryology, Xiangya School of Medicine, Central South University, Changsha 410011, China; ^5^State Key Laboratory of Pathogenesis, Prevention and Treatment of High Incidence Diseases in Central Asia, School of Pre-Clinical Medicine, Xinjiang Medical University, Urumqi, Xinjiang 86830011, China

## Abstract

**Objective:**

The aim of the present study was to investigate the effect of forkhead box M1 (FOXM1) to paclitaxel resistance in cervical cancer cells, to determine the underlying mechanism, and to identify novel targets for the treatment of paclitaxel-resistant cervical cancer.

**Methods:**

Paclitaxel-resistant Caski cells (Caski/Taxol cells) were established by intermittently exposing the Caski cells to gradually increasing concentrations of paclitaxel. The association between FOXM1, ATP-binding cassette subfamily C member 5 (ABCC5), and cervical cancer cell drug resistance was assessed by overexpressing or knocking down the expression of FOXM1 in Caski or Caski/Taxol cells. The protein and mRNA expression levels, the ratio of cellular apoptosis, and cell migration as well as intracellular drug concentrations were measured in cells following the different treatments.

**Results:**

After the successful establishment of resistant Caski/Taxol cells, cell cycle distribution analysis showed that a significantly larger percentage of Caski/Taxol cells was in the G0/G1 stage compared with the Caski cells (*P* < 0.01), whereas a significantly larger percentage of Caski cells was in the S and G2/M stage compared with the Caski/Taxol cells following treatment with paclitaxel (*P* < 0.01). Both the protein and mRNA expression levels of FOXM1 and ABCC5 transporters were significantly higher in the paclitaxel-resistant Caski/Taxol cells compared with Caski cells (*P* < 0.05). Knockdown of FOXM1 significantly lowered the protein expression levels of FOXM1 and ABCC5. Intracellular paclitaxel concentrations were significantly higher amongst the Caski/Taxol cells following the knockdown of FOXM1 by shRNA or Siomycin A (*P* < 0.05).

**Conclusion:**

FOXM1 promotes drug resistance in cervical cancer cells by regulating ABCC5 gene transcription. The knockdown of FOXM1 with shRNA or Siomycin A promotes paclitaxel-induced cell death by regulating ABCC5 gene transcription.

## 1. Introduction

Paclitaxel was approved by the US Food and Drug Administration for the treatment of ovarian cancer in 1992 and has since become a first-line treatment option for numerous types of cancer [1–3]. The primary target of paclitaxel is the intracellular microtubule system. By promoting microtubule polymerization and inhibiting microtubule depolymerization, paclitaxel can arrest cells in the G2/M phase, eventually resulting in cell death. During the initial treatment stages, most patients with cervical cancer show adequate sensitivity to chemotherapeutic drugs. However, following short-term treatment, acquired drug resistance may develop and result in failure of chemotherapy [4–6].

The molecular mechanism underlying chemoresistance to paclitaxel is not yet clear. It has been reported that the Fox family of molecules may induce paclitaxel resistance by upregulating BH3-interacting domain death agonist and BCL2 expression and activating the MAPK/JNK signaling pathway [7, 8]. Forkhead box M1 (FOXM1) is a transcription factor and a proliferation specific gene in the Fox family; its expression and transcription activity is vital in G1/S and G2/M cell cycle regulation, cell division, chromosome stability, and apoptosis [9, 10]. FOXM1 is upregulated in several types of cancer, and there is increasing evidence that FOXM1 is actively involved in tumor progression. In our previous studies, it was shown that the expression of FOXM1 is closely related to ATP-binding cassette (ABC) transporters, whose upregulation in cell membranes leads to increased drug efflux and decreased drug influx, which may be an important mechanism underlying the acquired resistance of cancers to drugs [11–13].

ATP-binding cassette subfamily C member 5 (ABCC5) is part of the multidrug resistance protein (MRP) family of multispecific drug transporters, in the C branch of the superfamily of ABC transporters. They work as drug efflux pumps to transport various molecules across cell membranes, and hyperactive extrusion of anticancer drugs leads to drug resistance. There are nine MRPs that have been identified in the human genome, including ABCC1-6 and ABCC10-12. ABCC5 is one of the critical ABC transporter molecules involved in paclitaxel drug resistance. In our previous study, it was shown that ABCC5 was overexpressed in paclitaxel-resistant nasopharyngeal carcinoma cells, and the expression levels were positively correlated with drug efflux and drug resistance. The knockdown of ABCC5 with small interfering (si)RNA significantly decreased drug efflux, thereby increasing the intracellular concentrations of paclitaxel to overcome paclitaxel drug resistance. Based on our previous studies, it was hypothesized that the FOXM1-ABCC5 axis contributes to paclitaxel resistance in cervical cancer cells, and this formed the subject of the present study, with the aim of identifying novel therapeutic targets to overcome paclitaxel resistance in cervical cancer cells.

## 2. Materials and Methods

The Caski cells were purchased from TONGPAI Biotechnology Co., Ltd. The paclitaxel-resistant Caski/Taxol cells were established by intermittently exposing the parental cells to gradually increasing concentrations of paclitaxel, as previously described [11, 14]. Cells were cultured in RPMI-1640 medium (Hyclone; Cytiva) containing 10% FBS (Gibco) with 100 U/ml penicillin and 100 *μ*g/ml streptomycin (Invitrogen; Thermo Fisher Scientific, Inc.).

### 2.1. Colony Formation Assay

Colony formation assay was performed in cells treated with stepwise concentrations of paclitaxel. To test the sensitivity of Caski and Caski/Taxol cells to paclitaxel, the cells were seeded in 6-well plates (1 × 10^3^ cells/well) and then cultured for 15 days to allow colony formation. The cell colonies were fixed in 4% paraformaldehyde for 15 min and stained by GIMSA (Sigma, 48900) for 30 min in room temperature. The dishes were imaged after staining. The cells were cleaned with 10% SDS, and the cell survival ratio was assessed by measuring the absorbance at 570 nm. Each treatment was performed in triplicate.

### 2.2. MTT Assay

Cells were cultured overnight in 96-well flat bottomed microtiter plates (5 × 10^3^ cells/well) and exposed to 0, 10, 20, 40, 80, 100, 200, or 250 *μ*M paclitaxel. After 0, 24, 48, or 72 h, 20 *μ*l MTT solution (Promega Corporation) was added to each well and cultured at 37°C in 5% CO_2_ for 4 h. A total of 100 *μ*l formazan solution was added to each well, and the cells were incubated at 37°C in 5% CO_2_ for 4 h. Absorbance at 570 nm was measured using a spectrometer. GraphPad Prism version 5 (GraphPad Software, Inc.) was used to assess the relative viability of the cancer cells using the following formula: [Control optical density (OD) − experimental OD]/Control OD. Each treatment was performed in quintuplicate.

### 2.3. Wound-Healing Assay

For wound-healing assays, Caski and Caski/Taxol cells were plated in 6-well plates (5 × 10^5^ cells/well) with RPMI-1640 (GIBCO, 11875093) cell culture medium containing 10% FBS (GIBCO, 16000-044) for 24 h. After cell adherence, the cells were washed with PBS three times. A confluent monolayer of cells was scratched using a 200 *μ*l plastic pipette tip. The cells were washed with PBS for three times and cultured with RPMI-1640 (GIBCO, 11875093) cell culture medium containing 1% FBS (GIBCO, 16000-044) [15]. Gaps between cells created were measured using the Image Pro Plus software (Media Cybernetics, Inc.) at 0 h, 12 h, 24 h, and 48 h after scratching. Cell migration in wound-healing assays was quantified using the following formula: (Cell gap at 0 h − cell gap at 12 h)/cell gap at 0 h × 100%.

### 2.4. Transwell Invasion Assay

For transwell invasion assays, Caski and Caski/Taxol cells were plated atop Matrigel-coated transwell chambers with 8 *μ*m pores (Costar Corp.) in serum-free media after being cultured in serum-free RPMI-1640 medium for 48 h. In the bottom chamber, media supplemented with 10% FBS was added. A total of 72 h after cell plating, the transwell chamber was extracted and fixed in 4% formaldehyde in room temperature for 20 min, washed with PBS twice, and put into well with 400 *μ*l Giemsa A solution for 1 min in room temperature; 800 *μ*l Giemsa solution was added into the well for 5 min; the transwell chamber was extracted and washed with PBS twice. The cells in the upper chamber were cleared using clean cotton tips, the lower chamber was dried and moved to slides, and three fields were observed under microscope, and the average number of cells was calculated. Each treatment was assessed in triplicate.

### 2.5. Flow Cytometry

Cell cycle distribution analysis was performed using a BD FACSCalibur flow cytometer (BD Biosciences). A total of 1 × 10^6^ Caski or Caski/Taxol cells were mixed with 5 ml 70% ethanol and kept at -20°C in the dark overnight. The following day, the cells were centrifuged at 1,000 rpm for 10 min, washed with PBS, and then suspended in 500 *μ*l PI/RNase Staining Buffer for 15 min at room temperature in the dark. The cells were filtered using 300 mesh filters before undergoing flow cytometry analysis and then analyzed by the ModFit LT V3.2 (Mac) software.

### 2.6. Preparation of Cells Up- or Downregulating FOXM1

Cells up- or downregulating FOXM1 were prepared lentiviral vectors encoding FOXM1 and FOXM1 shRNA. cDNA of FOXM1 was cloned into the pLV-EF1*α*-MCS-IRES-Bsd (Biosettia). The FOXM1 shRNA sequence: sense: 5′-GATCCGCTCTTCTCCCTCAGATATATTCAAGAGATATATCTGAGGGAGAAGAGTTTTTTG-3′ and anti-sense: 5′-AATTCAAAAAACTCTTCTCCCTCAGATATATCTCTTGAATATATCTGAGGGAGAAGAGCG-3′ was cloned into Lenti-X shRNA Expression Systems (Clontech Laboratories, Inc.). Nontarget shRNA (5′-TTCTCCGAACGTGTCACGT-3′) was used as the negative control.

Lentiviral vectors of FOXM1 and shRNA were cloned into 293T cells; the culture medium was changed 12 h later. Supernatant containing the lentivirus was harvested at 48 and 72 h to use for further experiments. When the cells reached 70-80% confluency, Caski/Taxol cells were infected with Lenti-X shRNA; Caski cells were infected with FOXM1 lentivirus. 48 h later, stable Caski/Taxol cells infected with FOXM1 shRNA lentivirus were selected with 2 *μ*g/ml puromycin, and stable Caski cells infected with FOXM1 lentivirus were selected with 8 *μ*g/ml BSD. Culture medium containing puromycin or BSD was changed 24 h later. The cells were passaged when reached 80% confluence. Cells were harvested for further experiments 2 weeks later.

### 2.7. RNA Extraction and Reverse Transcription-Quantitative (RT-q) PCR

The total RNA was extracted from cells using RNAiso Plus (Bio-Rad Laboratories, Inc.) according to the manufacturer's protocol. The dissolved RNA samples were measured on a spectrophotometer to determine the concentrations and quality prior to RT. qPCR was then performed using a CFX96TM Real-Time PCR Detection system (Bio-Rad Laboratories, Inc.) according to the manufacturer's protocol. The sequences of the primers used for qPCR were as follows: ABCC5 forward: 5′-AGTCCTGGGTATAGAAGTGTGAG-3′ and reverse: 5′-ATTCCAACGGTCGAGTTCTCC-3′; FOXM1 forward: 5′-GGAAGCAAAGGAGAAAACCC-3′ and reverse: 5-ATAGCAAGCGAGTCCGCATT-3′. The thermocycling conditions were as follows: initial denaturation at 95°C for 30 sec, followed by 40 cycles at 95°C for 5 sec and 60°C for 30 sec, with a final melt curve stage of 95°C for 15 sec, 60°C for 1 min, and 95°C for 15 sec. Values are expressed as fold changes compared with the corresponding values for the control using the 2-*ΔΔ*Cq method.

### 2.8. Western Blot Analysis

The cells were harvested, and total protein was extracted using RIPA lysis buffer. The protein samples (30-50 *μ*g) were loaded on an SDS-gel, resolved using SDS-PAGE, and transferred to a PVDF membrane (EMD Millipore). The membranes were blocked for 1 h with 5% nonfat milk dissolved in Tris-buffered saline with 0.1% Tween (TBS-T) and then incubated with the one of the following primary antibodies: anti-FOXM1 (1 : 500; Abcam, ab180710), GAPDH (1 : 500; Abcam, ab8245), or anti-ABCC5 (1 : 500; Abcam, ab180710) at 4°C overnight. Membranes were subsequently washed in TBS T three times and incubated for 1 h at room temperature with horseradish peroxidase-conjugated secondary antibodies (1 : 2,000; Santa Cruz Biotechnology, Inc.). Signals were visualized using a Pierce ECL Western Blotting Substrate detection system (Thermo Fisher Scientific, Inc.).

### 2.9. Luciferase Reporter Assay

The human ABCC5 gene promoter was cloned into a pGL3-TATA vector (Promega Corporation) to construct the ABCC5-luc vector. The ABCC5-luc vector and prl-sv40 luciferase reporter gene vector (Promega Corporation) were cotransfected with FoxM1 short hairpin (sh)RNA vector or FoxM1 overexpression vector using Lipofectamine® 2000 (Invitrogen; Thermo Fisher Scientific, Inc.). After 48 h, cells were collected and lysed using 1x ULB. Luciferase activity was detected using a Dual-Glo luciferase reporter assay system (Promega Corporation) according to the manufacturer's protocol 48 h after transfection. Fassay Substrate I was diluted to Fassay Reagent I with Rassay Buffer I at a ratio of 20 : 1; Fassay Substrate II was diluted to Fassay Reagent II with Rassay Buffer II at a ratio of 50 : 1. A total of 20 *μ*l cell lysate was mixed with 100 *μ*l Fassay Reagent I and 100 *μ*l Fassay Reagent II gently. The relative luciferase unit value of firefly/Renilla luciferase activities was measured using the PerkinElmer (EnSpire 2300) Multilabel Reader (PerkinElmer, Inc.).

### 2.10. ChIP and Quantitative Reverse-Transcriptase PCR Analysis

Caski and Caski/Taxol cells were prepared for the chromatin immunoprecipitation (ChIP) assay with the SimpleChIP® Sonication Chromatin IP kit: CST, #56383, according to the manufacturer's protocol. Briefly, for each ChIP, cells were isolated from two 10 cm plates. Cells were washed with phosphate-buffered saline (PBS) and incubated cells with 1% formalin in PBS for 10 min to crosslink proteins and DNA. Crosslinking was stopped with an incubation with 0.125 M glycine for 5 min. The cells were collected in ChIP Sonication Cell Lysis Buffer and sonicated to fragment genomic DNA into 200–1000 bp pieces. Aliquot of 5-10 *μ*g DNA fragments was diluted with ChIP dilution buffer until 500 *μ*l, 2% volume of chromatin was used as input, the rest were incubated with ChIP-specific antibody overnight at 4°C, and IgG antibody was used as control. G immunomagnetic beads were used to concentrate the antibody complex. The resulting precipitated DNA samples were analyzed using PCR to amplify a potential binding site region of the ABCC5 promoter with the primers 5′-CGGGTTAGACGCGGGCTACG-3′ (sense) and 5′-GCTGCCCCTCTTCCCACCGA-3′ (antisense). PCR products were resolved electrophoretically on a 2% agarose gel and visualized using ethidium bromide staining.

### 2.11. Drug Concentrations within the Cells

To test the sensitivity of Caski/Taxol cells to paclitaxel when FOXM1 expression was knocked down, Caski/Taxol cells were first transfected with FOXM1 shRNA for 24 h or treated with Siomycin A (Calbiochem; Merck KGaA) for 48 h. The cells were then treated with paclitaxel (80 *μ*M) marked with 10 mM fluorescent for 48 h and stained with Oregon Green™ 488 Conjugate (Oregon Green™ 488 Taxol, Flutax-2, Thermo Fisher Scientific, Inc.; cat. no. P22310) for 24 h before analyzing using flow cytometry (BD, FACSCalibur). Cells were fixed on a glass slide and stained with DAPI before being observed by confocal laser scanning microscopy (Leica Microsystems, Inc.) to assess fluorescence in the cytoplasm and nuclei.

### 2.12. Statistical Analysis

All in vitro experiments were performed either in triplicate or in quintuplicate. Statistical analysis was performed using SPSS version 24.0 (IBM Corp.). Two-sided Student's *t*-tests were used for comparison of different parameters between the two groups. Data were presented as the mean ± the standard deviation. *P* < 0.05 was considered to indicate a statistically significant difference.

## 3. Results

By applying intermittent low doses of paclitaxel, a paclitaxel-resistant NPC cell line was established in our previous studies, and this method was used in the present study to develop Caski human cervical carcinoma cells that were resistant to paclitaxel, which were termed Caski/Taxol cells [11, 14]. Chemotherapeutic resistance of Caski and Caski/Taxol cells was assessed by treating cells with an IC50 dose of paclitaxel and then using an MTT assay. Paclitaxel (50, 100, 150, 200, and 250 *μ*M) significantly reduced the viability of Caski cells compared with the Caski/Taxol cells 48 h after treatment (Figures 1(a) and 1(b)). The IC50 was 50.55 *μ*M (95% confidence interval (CI), 39.95-63.97) for Caski cells and 88.82 *μ*M (95% CI, 79.92-98.70) for Caski/Taxol cells (*P* < 0.01; Figure 1(b)). Cell cycle distribution of Caski and Caski/Taxol cells was assessed using PI fluorescence with a BD FACSCalibur flow cytometry and analyzed using the ModFit analytic software. Cell cycle analysis showed that 74.7% of Caski/Taxol cells were in the G0/G1 stage, compared with 49.8% of Caski cells (*P* < 0.01). Meanwhile, 15.9 and 9.4% of Caski/Taxol cells were in the S and G2/M stages, compared with 32.2 and 18.0% of Caski cells, respectively (*P* < 0.01; Figure 1(c)).

### 3.1. Cell Migration and Invasion Tests

Paclitaxel-resistant Caski cells exhibit increased migration and invasion. Based on the results of the wound-healing assay, migration was significantly increased in the Caski/Taxol cells compared with the Caski cells (Figure 2(a)). In the transwell cell invasion assays, invasion was significantly increased in the Caski/Taxol cells compared with the Caski cells (Figure 2(b)).

### 3.2. Intracellular Drug Concentrations

To further evaluate the resistance of Caski/Taxol cells to paclitaxel, the intracellular drug concentrations were measured in the Caski/Taxol and Caski cells. Caski/Taxol and Caski cells were treated with 80 *μ*M Flutax-2 for 48 h, and intracellular green fluorescence was monitored by confocal microscopy (Figure 3(a)), and the strength of fluorescence was measured using flow cytometry (Figure 3(b)). The results showed that fluorescence in Caski/Taxol cells was significantly weaker compared with that in Caski cells, indicating significantly lower intracellular drug concentrations of paclitaxel in the Caski/Taxol cells compared with the Caski cells.

### 3.3. Effect of FOXM1 and ABCC5 on Caski and Caski/Taxol Cells

FOXM1 and ABCC5 transporter expression is significantly increased in the Caski/Taxol cells compared with the Caski cells. FOXM1 primarily regulates G1/S phase and G2/M phase transitions via modulation of cell cycle regulatory genes, and ABCC5 has been reported to be a target. In our previous studies, it was shown that FOXM1 enhances chemoresistance via regulating ABCC5 gene transcription in NPC cells by binding to the FHK consensus motif in the promoter region of the ABCC5 gene [11]. Combining the significant increase in paclitaxel efflux in Caski/Taxol cells with our previous findings, it was hypothesized that the paclitaxel resistance may be caused by the FOXM1-mediated ABCC5 elevation. When comparing the protein and mRNA expression levels of FOXM1 and ABCC5 in Caski/Taxol and Caski cells, significantly higher expression levels of both FOXM1 and ABCC5 were detected in the Caski/Taxol cells compared with the Caski cells at both the protein and mRNA levels (Figures 4(a) and 4(b)). The association between FOXM1 and ABCC5 was assessed by determining the effect on ABC transporters following the knockdown of FOXM1. shRNA-mediated FOXM1 knockdown significantly lowered the protein expression levels of FOXM1 and ABCC5 (Figure 4(c)). The luciferase activity of the ABCC5 gene promoter was assessed when the Caski/Taxol cells were cotransfected with an ABCC5 gene promoter, a FOXM1 promoter, or a FOXM1 inhibitor. The expression of the ABCC5 gene promoter increased following FOXM1 overexpression and decreased following FOXM1 inhibition (Figure 4(d)), further indicating a positive association between FOXM1 and ABCC5. Caski/Taxol cells were prepared for the ChIP assay using a SimpleChIP® Sonication Chromatin IP kit. The results of the ChIP experiments showed that the binding of FOXM1 to the FHK consensus motif in the ABCC5 gene promoter was significantly higher in the Caski/Taxol cells compared with *β*-actin (Figure 4(e)).

Intracellular paclitaxel concentrations were measured using confocal microscopy (Figures 5(a) and 5(c)) and flow cytometry (Figures 5(b) and 5(d)) following treatment of the Caski/Taxol cells with Flutax-2 for 48 h after knockdown of FOXM1 by shRNA (Figure 5(a)or 5(b)) or Siomycin A (Figures 5(c) and 5(d)). The results showed that intracellular paclitaxel concentrations were significantly increased following FOXM1 downregulation by both shRNA and Siomycin A, indicating the potential of Siomycin A in sensitizing chemo-resistant cancer cells to paclitaxel.

## 4. Discussion

Cancer drug resistance is primarily the result of abnormalities in drug transportation and metabolism, which could be caused by mutations of target genes, abnormal DNA repair, decreased tumor apoptosis, cell aging, autophagy, and changes in the tumor microenvironment [16–18]. FOXM1 interacts with a variety of oncogenes and tumor suppressor genes and participates in multiple signal transduction pathways, several of which are closely related to drug resistance. However, the mechanism by which FOXM1 increases resistance to paclitaxel in cervical cancer has not been fully elucidated [19, 20].

At present, one of the primary methods to restore the sensitivity of drug-resistant cancer cells to chemotherapeutic drugs is by inhibiting the expression or function of transporters. ABC transporters are a group of transmembrane proteins. They have a one-way substrate transport pump and an ATP-binding region and actively carry out the transmembrane transport of various molecules. According to sequence homology and transmembrane topological structure analysis, ABC transporters are divided into seven subfamilies (ABCA-ABCG). Proteins in the ABCC subfamily are closely involved in mediating drug transport [6]. Amongst the nine primary transporters (ABCC1-6, ABCC10-12, or MRP 1-9) in the ABCC family, ABCC5 was found to transport nucleoside monophosphate analogues and produce cancer drug resistance [21–23].

FOXM1 is a transcription factor in the FOX family that regulates cellular proliferation, apoptosis, and chromosomal stability. FOXM1 was found to be upregulated in various tumor lesions [24, 25]. The significance of the FOXM1-ABCC5 axis in paclitaxel resistance in NPC cells was shown in our previous study [11]. The present study assessed whether resistance to paclitaxel was increased following upregulation of FOXM1 and ABCC5 in cervical cancer cells. Following the establishment of the Caski/Taxol cells, paclitaxel-induced cell death was assessed by treating cells with an IC50 dose of paclitaxel and performing an MTT assay. The results showed a significant decrease in cell viability in the Caski cells compared with the Caski/Taxol cells following treatment with any dosage of paclitaxel for 48 h, demonstrating the establishment of the paclitaxel-resistant Caski/Taxol cell line. Cell migration assays also showed significantly increased migration in the Caski/Taxol cells compared with the Caski cells 48 h after creating the wound. Similarly, the transwell invasion assays showed increased invasion in the Caski/Taxol cells compared with the Caski cells. Together, these results showed successful establishment of a paclitaxel-resistant cervical cancer cell line, which was termed Caski/Taxol. Next, the Caski/Taxol cells were treated with paclitaxel for 24 h, which resulted in a significant increase in FOXM1 and ABCC5 in the Caski/Taxol cells, and ABCC5 expression was decreased following knockdown of FOXM1, leading to increased intracellular drug concentrations. In our previous study, we proved that FOXM1 promotes drug resistance in nasopharyngeal carcinoma cells by regulating ABCC5 gene transcription. The current study is the extension of our previous study and found that the ratio of cellular apoptosis and cell migration as well as intracellular drug concentrations can be controlled by overexpressing or knocking down the expression of FOXM1, providing FOXM1 as a target for the treatment of cervical cancer that is resistant to paclitaxel.

The results of the present study combined with the results of previous studies showed that FOXM1 promotes drug resistance to paclitaxel by increasing the expression of ABCC5. To the best of our knowledge, the present study is the first to show that FOXM1 regulated drug efflux and paclitaxel resistance via modulation of gene transcription of ABCC5 in cervical cancer cells. The results highlight potentially novel therapeutic targets and novel approaches for the management of paclitaxel-resistant cervical cancer. In the meanwhile, although we established the new cervical cancer drug-resistant cell line in the current study, we have only tested paclitaxel and did not test other cancer drugs such as 5-FU. Our future studies will be concentrated on the other anticancer drugs. Now, it is mentioned in Introduction and Discussion. Moreover, previous studies have reported that paclitaxel is an excellent P-glycoprotein (ABCB1) substrate [26, 27], and that multidrug resistance-associated protein 7 (MRP7/ABCC10) expression is a predictive biomarker for the resistance to paclitaxel in various types of cancer cells [28–30]. Further studies should be carried out to test if paclitaxel resistance in cervical cancer cells relate to the expression of P-gp or MRP7/ABCC10.

In conclusion, FOXM1 may promote drug resistance in cervical cancer cells by regulating ABCC5 gene transcription. The depletion of FOXM1 with shRNA or Siomycin A can block drug efflux and increase the intracellular concentrations of paclitaxel, thereby promoting paclitaxel-induced cell death.

## Figures and Tables

**Figure 1:** (a) Colony formation assay of Caski and Caski/Taxol cells cultured with 80 *μ*M paclitaxel for 48 h. Magnification, 400x. (b) IC50 dose of paclitaxel for Caski cells was 50.55 *μ*M (95% CI, 39.95-63.97) and 88.82 *μ*M (95% CI, 79.92-98.70) for Caski/Taxol cells. The Caski/Taxol cells exhibited significantly increased viability when treated with paclitaxel compared with the Caski cells. (c) Cell cycle distribution analysis showed that 74.7% cells of Caski/Taxol cells were in the G0/G1 stage, compared with 49.81% of the Caski cells. Additionally, 15.94 and 9.36% of Caski/Taxol cells were in the S and G2/M stages, compared with 32.24 and 17.95% of Caski cells. ^∗∗^Compared with Caski cells: *P* < 0.01. Caski/Taxol: paclitaxel-resistant Caski cells; CI: confidence interval.

**Figure 2:** (a) Wound-healing assays showed significantly increased migration in the Caski/Taxol cells compared with the Caski cells at 12 h, 24 h, and 48 h after scratching. (b) Transwell invasion assays also showed increased invasion by Caski/Taxol cells compared with the Caski cells after 72 h; ^∗∗^*P* < 0.01. Caski/Taxol: paclitaxel-resistant Caski cells.

**Figure 3:** (a) Intracellular green fluorescence was monitored by confocal microscopy, and (b) the strength of fluorescence was measured by flow cytometry. The results showed that fluorescence in the Caski/Taxol cells was significantly weaker compared with that in the Caski cells, indicating significantly lower intracellular drug concentrations of paclitaxel in the Caski/Taxol cells. ^∗∗^*P* < 0.01. Caski/Taxol: paclitaxel-resistant Caski cells.

**Figure 4:** FOXM1 and ABCC5 transporter expression is significantly increased in the Caski/Taxol cells compared with the Caski cells. (a) Protein and (b) mRNA expression levels of FOXM1 and ABCC5 were consistently significantly increased in the Caski/Taxol cells compared with the Caski cells. ^∗∗^*P* < 0.01 and ^∗∗∗^*P* < 0.001 vs. Caski cells. (c, d) FOXM1 knockdown significantly lowered the protein expression levels of FOXM1 and ABCC5, indicating a positive correlation between FOXM1 and ABCC5. ^∗∗^*P* < 0.01 vs. empty vector group. (e) ChIP analysis showed that the binding of FOXM1 to the FHK consensus motif of the abcc5 gene promoter was weak in the Caski cells, whereas in the paclitaxel-resistant Caski/Taxol cells, this binding was much stronger. ChIP: chromatin immunoprecipitation; Caski/Taxol: paclitaxel-resistant Caski cells; FOXM1: forkhead box M1; ABCC5: ATP-binding cassette subfamily C member 5.

**Figure 5:** Intracellular paclitaxel concentrations were measured by (a, c) confocal microscopy and (b, d) flow cytometry after treating the Caski/Taxol cells with 80 *μ*M Flutax-2 for 48 h following the knockdown of FOXM1 using (a, b) shRNAs or (c, d) inhibition of FOXM1 using Siomycin A. The results showed that intracellular paclitaxel concentrations were significantly increased following FOXM1 knockdown by shRNA or inhibition by Siomycin A, indicating the potential of Siomycin A to sensitize chemo-resistant cancer cells to paclitaxel. ^∗∗∗^*P* < 0.001. Caski/Taxol: paclitaxel-resistant Caski cells; shRNA: small interfering RNA; FOXM1: forkhead box M1.

## Data Availability

Data is available from the corresponding author upon request.

## References

[1] Yang Y. H., Mao J. W., Tan X. L. (2020). Research progress on the source, production, and anti-cancer mechanisms of paclitaxel. *Chinese Journal of Natural Medicines*.

[2] Lau T. S., Chan L. K. Y., Man G. C. W. (2020). Paclitaxel induces immunogenic cell death in ovarian cancer via TLR4/IKK2/SNARE-dependent exocytosis. *Cancer Immunology Research*.

[3] Zhu L., Chen L. (2019). Progress in research on paclitaxel and tumor immunotherapy. *Cellular & Molecular Biology Letters*.

[4] Miyamoto M., Sawada K., Nakamura K. (2020). Paclitaxel exposure downregulates miR-522 expression and its downregulation induces paclitaxel resistance in ovarian cancer cells. *Scientific Reports*.

[5] Meng X., Laidler L. L., Kosmacek E. A. (2013). Induction of mitotic cell death by overriding G2/M checkpoint in endometrial cancer cells with non-functional p53. *Gynecologic Oncology*.

[6] Němcová-Fürstová V., Kopperová D., Balušíková K. (2016). Characterization of acquired paclitaxel resistance of breast cancer cells and involvement of ABC transporters. *Toxicology and Applied Pharmacology*.

[7] Khan N., Kahl B. (2018). Targeting BCL-2 in hematologic malignancies. *Targeted Oncology*.

[8] Yu-Wei D., Li Z. S., Xiong S. M. (2020). Paclitaxel induces apoptosis through the TAK1-JNK activation pathway. *FEBS Open Bio*.

[9] Gartel A. L. (2017). FOXM1 in cancer: interactions and vulnerabilities. *Cancer Research*.

[10] Shibui Y., Kohashi K., Tamaki A. (2021). The forkhead box M1 (FOXM1) expression and antitumor effect of FOXM1 inhibition in malignant rhabdoid tumor. *Journal of Cancer Research and Clinical Oncology*.

[11] Hou Y., Zhu Q., Li Z. (2017). The FOXM1-ABCC5 axis contributes to paclitaxel resistance in nasopharyngeal carcinoma cells. *Cell Death & Disease*.

[12] Zhu X., Xue L., Yao Y. (2018). The FoxM1-ABCC4 axis mediates carboplatin resistance in human retinoblastoma Y-79 cells. *Acta Biochimica et Biophysica Sinica*.

[13] Xie T., Geng J., Wang Y. (2017). FOXM1 evokes 5-fluorouracil resistance in colorectal cancer depending on ABCC10. *Oncotarget*.

[14] Zhou Z., Zhang L., Xie B. (2015). FOXC2 promotes chemoresistance in nasopharyngeal carcinomas via induction of epithelial mesenchymal transition. *Cancer Letters*.

[15] Wang Y. F., Yang H. Y., Shi X. Q., Wang Y. (2018). Upregulation of microRNA-129-5p inhibits cell invasion, migration and tumor angiogenesis by inhibiting ZIC2 via downregulation of the Hedgehog signaling pathway in cervical cancer. *Cancer Biology & Therapy*.

[16] Panda M., Biswal B. K. (2019). Cell signaling and cancer: a mechanistic insight into drug resistance. *Molecular Biology Reports*.

[17] Haider T., Pandey V., Banjare N., Gupta P. N., Soni V. (2020). Drug resistance in cancer: mechanisms and tackling strategies. *Pharmacological Reports*.

[18] Mansoori B., Mohammadi A., Davudian S., Shirjang S., Baradaran B. (2017). The different mechanisms of cancer drug resistance: a brief review. *Advanced Pharmaceutical Bulletin*.

[19] Yao S., Fan L. Y., Lam E. W. (2018). The FOXO3-FOXM1 axis: a key cancer drug target and a modulator of cancer drug resistance. *Seminars in Cancer Biology*.

[20] Nandi D., Cheema P. S., Jaiswal N., Nag A. (2018). FoxM1: repurposing an oncogene as a biomarker. *Seminars in Cancer Biology*.

[21] Robey R. W., Pluchino K. M., Hall M. D., Fojo A. T., Bates S. E., Gottesman M. M. (2018). Revisiting the role of ABC transporters in multidrug-resistant cancer. *Nature Reviews. Cancer*.

[22] Amawi H., Sim H. M., Tiwari A. K., Ambudkar S. V., Shukla S. (2019). ABC transporter-mediated multidrug-resistant cancer. *Advances in Experimental Medicine and Biology*.

[23] Chen J., Wang Z., Gao S. (2021). Human drug efflux transporter ABCC5 confers acquired resistance to pemetrexed in breast cancer. *Cancer Cell International*.

[24] Zhu X., Lu K., Cao L., Hu Y., Yin Y., Cai Y. (2020). FoxM1 is upregulated in osteosarcoma and inhibition of FoxM1 decreases osteosarcoma cell proliferation, migration, and invasion. *Cancer Management and Research*.

[25] Barger C. J., Branick C., Chee L., Karpf A. R. (2019). Pan-cancer analyses reveal genomic features of FOXM1 overexpression in cancer. *Cancers*.

[26] Alam A., Kowal J., Broude E., Roninson I., Locher K. P. (2019). Structural insight into substrate and inhibitor discrimination by human P-glycoprotein. *Science*.

[27] Jang S. H., Wientjes M. G., Au J. L. S. (2001). Kinetics of P-glycoprotein-mediated efflux of paclitaxel. *Journal of Pharmacology and Experimental Therapeutics*.

[28] Zhou Y., Hopper-Borge E., Shen T. (2009). Cepharanthine is a potent reversal agent for MRP7(ABCC10)-mediated multidrug resistance. *Biochemical Pharmacology*.

[29] Oguri T., Ozasa H., Uemura T. (2008). MRP7/ABCC10 expression is a predictive biomarker for the resistance to paclitaxel in non-small cell lung cancer. *Molecular Cancer Therapeutics*.

[30] Wang J. Q., Wang B., Teng Q. X. (2021). CMP25, a synthetic new agent, targets multidrug resistance-associated protein 7 (MRP7/ABCC10). *Biochemical Pharmacology*.

